The article "Senkyunolide H Affects Cerebral Ischemic Injury through Regulation on Autophagy of Neuronal Cells via P13K/AKT/mTOR Signaling Pathway" was retracted in 2023. Reasons: unreliable results or conclusions; concerns about the data; concerns about the peer review; concerns about the citations.

# Senkyunolide H Affects Cerebral Ischemic Injury through Regulation on Autophagy of Neuronal Cells via P13K/AKT/mTOR Signaling Pathway

**DOI:** 10.1155/2022/9211621

**Published:** 2022-10-03

**Authors:** Bei Zhao, Ke-Cheng Tang, Ying Zhao, Wang Zhao

**Affiliations:** ^1^Department of Neurology, The Affiliated Hospital of Inner Mongolia Medical University, Hohhot, 010030 Inner Mongolia, China; ^2^Department of General Surgery, The Second Affiliated Hospital of Inner Mongolia Medical University, Hohhot, 010030 Inner Mongolia, China; ^3^Department of Laboratory, Shanghai Xuhui District Dahua Hospital, Shanghai 200231, China; ^4^Department of Neurology, Yongchuan Hospital of Chongqing Medical University, Chongqing Key Laboratory of Cerebrovascular Disease Research, Chongqing 402160, China

## Abstract

Cerebral ischemia (CI) is associated with high global incidence and risk; therefore, its rapid and reliable therapeutic management is essential for protecting patients' lives and improving health. Senkyunolide H (SH) is remarkably effective against phlebosclerosis, oxidation, and apoptosis. Blood-brain barrier is the main obstacle impeding the delivery of drugs and xenobiotics to brain areas. Drugs' loading in nanoparticles can overcome the blood-brain barrier obstacle and thus directly and completely act on brain tissue, and such a loading can also change the half-life of drugs *in vivo* and lower the dosage requirement of drugs. In this study, we loaded the SH in lipid nanoparticles to improve its delivery to the brain for the therapy of CI. Thus, this study preliminarily analyzed the mechanism of SH-loaded nanoparticles in CI. The SH-loaded lipid nanoparticles were prepared and characterized with electron microscopy and PS potentiometery. The SH-loaded nanoparticles were intraperitoneally administered to CI-induced rats and brain tissue water content, and neuronal apoptosis and autophagy-associated proteins were determined. Our assays revealed SH-loaded nanoparticle's ability to reduce nerve injury and brain tissue water content in rats with CI and inhibit the apoptosis and autophagy of their neuronal cells (NCs). Additionally, under intervention with SH-loaded nanoparticles, P13K/AKT/mTOR pathway-associated proteins in brain tissue of rats decreased. As the assay results showed, SH-loaded nanoparticles can suppress the autophagy of NCs through medicating P13K/AKT/mTOR pathway and lower apoptosis, thus delivering the effect of treating CI. Results of this study indicate SH-loaded nanoparticles as promising strategy for delivery SH to brain areas for treating CI.

## 1. Introduction

Cardio-cerebrovascular diseases and chronic diseases with the highest global incidence are frequent among middle-aged and aged population [1]. Cerebral ischemia (CI) is a commonly occurring disease in elderly posing enormous threat to heath of the elder population [2]. Its occurrence is probably induced by atherosclerosis, hypertension, thrombosis, hyperlipidemia, diabetes, excitement, fatigue, and many others [3]. Without timely and effective therapy, CI might directly induce cerebral infarction, giving rise to irreversible neurological function deficit and even endanger patients' life and health in severe cases [4]. Currently, over 20 million new cases of CI are observed each year worldwide, and the number goes up annually as the global rate of elder population increases [5, 6]. Conservative therapy is preferred for the management of CI, where medicines are prescribed to the patients for a long run to control CI attack [7]. For CI with multiple and complex inducements, effective plan to completely cure is still under investigation [8]. Thus, researchers are constantly searching to find out an efficient and effective way against CI [9].

The article "Senkyunolide H Affects Cerebral Ischemic Injury through Regulation on Autophagy of Neuronal Cells via P13K/AKT/mTOR Signaling Pathway" was retracted in 2023. Reasons: unreliable results or conclusions; concerns about the data; concerns about the peer review; concerns about the citations.

Earlier studies have shown a strong link of CI with biological behavior changes of neuronal cells (NCs) many times [10, 11]. Autophagy, a physiological process of cell metabolism, plays a crucial role in the development of many diseases [12, 13]. Among cases with CI, autophagy of NCs can notably accelerate their apoptosis and thereby give rise to nerve tissue injury [14].

Ligusticum chuanxiong, a natural Chinese medicine component, is most frequently adopted as a medicine for promoting blood circulation and removing blood stasis [15]. Senkyunolide H (SH) is a typical phenolic compound found in Ligusticum chuanxiong. It has been shown to have remarkable effects against phlebosclerosis, oxidation, and apoptosis and in regulating inflammatory response [16]. However, during the development of CI, blood-brain barrier is highly prone to prevent the drug reaction from entering the brain tissue [17]. Loading drugs in nanoparticles are an advancement in the field of drug delivery where the drugs are converted to nanosized particles and improve its bioavailability. Drugs within nanoparticles with extremely small molecular structure and high activity as carriers can be delivered to various tissues and organs in the human body quickly [18]. In addition, nanoparticles can change the half-life of drugs *in vivo* and lower the dosage requirement of drugs [19]. Nanocarrier-based drugs have also been shown to traverse the blood-brain barrier and successfully deliver the loaded drug into brain areas. Therefore, we designed this study to prepare SH-loaded lipid nanoparticles and investigate its delivery to the brain for improving the current treatment status of CI and analyze its impact on CI and associated mechanisms, with the aim of offering novel reference of clinical therapy of CI.

The article "Senkyunolide H Affects Cerebral Ischemic Injury through Regulation on Autophagy of Neuronal Cells via P13K/AKT/mTOR Signaling Pathway" was retracted in 2023. Reasons: unreliable results or conclusions; concerns about the data; concerns about the peer review; concerns about the citations.

## 2. Materials and Methods

### 2.1. Experimental Animal Data

Thirty Wistar rats (3-6 months old weighing 200-250 g) were purchased from Shanghai Medicilon Biopharmaceutical Co., Ltd. (animal license: SYXK (Shanghai) 2020-0038) and housed under 25°C and 40% humidity, with free access to light and drinking water. The study was conducted in Department of Neurology, Yongchuan Hospital of Chongqing Medical University, Chongqing, China. The flowchart of the study was shown in Figure 1.

### 2.2. Modeling Methods

The rats were randomly assigned to three groups. One group was kept as control and fed normally without any intervention, and the other two groups' animals were spared for CI modeling. Specifically, with reference to one study by Haji et al. [20], rats were anesthetized through intraperitoneal injection of 1% pentobarbital sodium (40 mg/kg), then immobilized in prone position, and routinely disinfected the head and hairs from the top of head that were removed. Then, a high-frequency electrotome was used for blocking the vertebral artery flow in left and right transverse foramina of the transverse process wings of the first cervical vertebra of each rat. After 24 h, the bilateral common carotid arteries were clamped by arterial clamp for 5 min. After modeling, rats with obvious confusion of consciousness, dilated pupils, shortness of breath, decreased pain, and no response of pupils to light source were regarded as successfully modeled.

### 2.3. Neurological Deficit Score (NDS) of Rats

The neurological function deficiency of the animals was assessed by an adopted scale where no signs: 0 points; inability of completely straightening the forelimb: 1 point; paralysis of one limb: 2 points; inability of standing up: 3 points; and no spontaneous activity: 4 points.

### 2.4. Detection of Brain Injury Markers

Blood from tail veins of the animals (0.5 mL) was subjected to 10 min centrifugation (1509 × g, 4°C) for serum collection, followed by determination of serum neuron-specific enolase (NES) and S-100*β* via enzyme linked immunosorbent assay (ELISA).

### 2.5. Preparation of SH-Loaded Nanoparticles

Dioleoyl lecithin (15 mg), cholesterol (5 mg), and distearate phosphatidylethanolamine-polyethylene glycol 2000 (15 mg) were dissolved in 30 mL chloroform and mixed thoroughly. Dioleoyl lecithin, cholesterol, distearate phosphatidylethanolamine-polyethylene glycol 2000, and chloroform were all purchased from Sigma-Aldrich via local supplier (the chemicals and solvents used in this study were of analytical grade and used as such without further purification). The organic solvent was removed by rotary evaporation (37°C) until dryness, and a film-like substance was formed on the base of the rotary flask. The film was dried for 12 h in a vacuum box, followed by addition of SH (15 mg) in 0.01 M preheated PBS. Finally, the mix was given 2 h centrifugation (500 × g, 37°C) and filtering via 0.22 *μ* L filter membrane, followed by dying (4°C) to prepare SH-loaded nanoparticles.

The article "Senkyunolide H Affects Cerebral Ischemic Injury through Regulation on Autophagy of Neuronal Cells via P13K/AKT/mTOR Signaling Pathway" was retracted in 2023. Reasons: unreliable results or conclusions; concerns about the data; concerns about the peer review; concerns about the citations.

### 2.6. Establishment of Standard Curve of SH-Loaded Nanoparticles

SH-loaded nanoparticles (1 mg) were dissolved in methanol (1 mL) and serially diluted to 2.5, 5, 10, 20, 30, and 40 *μ*g*/*mL with methanol. The absorption of all the solutions was measured using the HPLC system (Shimadzu, Kyoto, Japan), and a standard curve was established.

### 2.7. Characterization of SH-Loaded Nanoparticles

The morphology of nanoparticles was observed under scanning electron microscope, and the particle size distribution was analyzed by nanosize potentiometer.

### 2.8. Intervention of SH-Loaded Nanoparticles on Rats with CI

Among the two groups of model rats, one group was intervened with SH-loaded nanoparticles as an SH group where the rats were administered 50 mg/kg SH-loaded nanoparticles 2 h after modeling. The other group was intervened with the same amount of normal saline as a model group (Mod group). Administration of both groups was completed within 24 h.

### 2.9. Determination of Brain Tissue Water Content (BTWC)

The rats were euthanized by cervical dislocation under anesthesia, and their brains were taken and cut open along the coronal plane of the pinhole. A slice (approximate 3 mm thick) was taken in front of the pinhole, and the blood and cerebrospinal fluid were sucked off. The wet weight was measured by electronic balance. Then, the brain was subjected to 24 h drying (95**°**C) in an incubator, followed by measurement of dry weight. The water content in the brain tissue was determined by the formula below:

(1) $$\begin{array}{c} \text{Water content }\left(\%\right)=\left(\text{wet weight}-\text{dry weight}\right)\left(\text{g}\right)/\text{wet weight }\left(\text{g}\right)\times 100\% \end{array}$$

### 2.10. Determination of Neuronal Apoptosis

Single-cell suspension (1 × 10^6^ cells/mL) was prepared from brain tissue (30-50 mg), followed by 10 min reaction with 1 *μ*L Annexin-V-FITC and 5 *μ*L propidium iodid (PI) under dark environment and then addition of 400 *μ*L buffer. Finally, flow cytometry was performed for determination of cell apoptosis.

### 2.11. Detection of Autophagy-Associated Proteins in NCs

Brain tissue of rats was lysed, followed by treatment with SDS-PAGE and transfer to a membrane. The tissue was overnight incubated (4**°**C) after being diluted with Tris-buffered saline with Tween-20 (0.1%) (TBST) to 1 : 1000 on a shaking bath. After being cleaned via TBST, second antibody was put in. One hour later, the gray value was evaluated via a BCA protein quantitative kit (Beyotime Biotechnology; Shanghai).

The article "Senkyunolide H Affects Cerebral Ischemic Injury through Regulation on Autophagy of Neuronal Cells via P13K/AKT/mTOR Signaling Pathway" was retracted in 2023. Reasons: unreliable results or conclusions; concerns about the data; concerns about the peer review; concerns about the citations.

### 2.12. Statistical Analyses

SPSS (Version 22.0; IBM, US) was used for statistical analysis. Results were recorded as mean ± SD and analyzed via independent-samples *t*-test, one-way ANOVA, LSD test, repeated variance, or Bonferroni test. *P* < 0.05 was considered as statistically significant difference.

## 3. Results

### 3.1. Modeling Results of Rats with CI

Modeling results of rats with CI are shown in Figure 2.  Figure 2(a) shows nerve defect score of the model rat with the control group representing that the model rats' nerve defect was statistically significant.  Figure 2(b) shows serum neuron-specific enolase (NES) concentration of the model rat in comparison with the control group suggesting that the concentration of NES was high in the model rat group.  Figure 2(c) depicts S-100*β* concentration of the model rat and control groups suggesting that S-100*β* concentration was high in the model rat group. The Mod group got a notable higher NDS than the control group (Con group) (2.87 ± 0.67) points vs. (1.00 ± 0.47) points, (*P* < 0.05, Figure 2(a)) and showed NES and S-100*β* of 22.68 ± 2.83 pg/mL and 242.15 ± 17.64 ng/mL, respectively, both notably higher than those in the Con group (both *P* < 0.05, Figures 2(b) and 2(c)).

### 3.2. Preparation Results of SH-Loaded Nanoparticles

After determination of the peak areas under different concentrations of SH-loaded nanoparticle solutions, a standard curve of SH-loaded nanoparticles was constructed with drug concentration of SH-loaded nanoparticles as the ordinate and the peak area as the abscissa (Figures 3(a) and 3(b)).

### 3.3. Characterization of SH-Loaded Nanoparticles

Under the electron microscope, SH-loaded nanoparticles showed even distribution and densely round structure, with obvious substances in the gaps between the particles that might be free SH (Figure 4(a)), and indicated SH-loaded nanoparticles obtained good shape and size distribution uniformity with fewer impurity content. According to the PS spectrometer, the PS of SH-loaded nanoparticles was around 80-120 nm (Figure 4(b)).

### 3.4. Impact of SH-Loaded Nanoparticles on NDS of Rats

The SH group showed neurological deficit score (NDS) of (1.84 ± 0.52) points, lower than that of the Mod group, but higher than that of the Con group (*P* < 0.05, Figure 5).

The article "Senkyunolide H Affects Cerebral Ischemic Injury through Regulation on Autophagy of Neuronal Cells via P13K/AKT/mTOR Signaling Pathway" was retracted in 2023. Reasons: unreliable results or conclusions; concerns about the data; concerns about the peer review; concerns about the citations.

### 3.5. Impact of SH-Loaded Nanoparticles on Nerve Injury

The SH group showed NES and S-100*β* concentrations of (15.63 ± 1.18) pg/mL and (192.66 ± 8.42) ng/mL, lower than those in the Mod group, but higher than those in the Con group (all *P* < 0.05, Figures 6(a) and 6(b)). Additionally, the SH group had BTWC of (74.33 ± 4.24) %, which was also lower than that of the Mod group, but higher than that of the Con group (*P* < 0.05, Figure 6(c)).

### 3.6. Impact of SH-Loaded Nanoparticles on Neuronal Apoptosis

Compared to the control group, the apoptosis rate in the model group was significantly increased; after SH-loaded nanoparticles intervention on rats with CI, the apoptosis rate was decreased. Bcl-2 and Bax are a pair of homologous genes regulating cell apoptosis. The high expression of Bcl-2 can inhibit the occurrence of cell apoptosis, and Bax can antagonize the antiapoptotic effect of Bcl-2 and play a role in accelerating cell apoptosis.The SH group showed higher protein expression of Bcl-2 and lower protein expression of Bax than the model group and the control group (all *P* < 0.05, Figures 7(a) and 7(b)).

### 3.7. Impact of SH-Loaded Nanoparticles on Autophagy of NCs

The SH group had no difference in Beclin-1 and LC3 when compared with the control group but showed lower levels of Beclin-1 and LC3 when compared with the model group (all *P* < 0.05, Figure 8).

### 3.8. Impact of SH-Loaded Nanoparticles on P13K/AKT/mTOR Pathway

The SH group animals showed lower levels of P13K, AKT, and mTOR than the model group and higher levels of P13K, AKT, and mTOR when compared with the control group (all *P* < 0.05, Figure 9).

## 4. Discussion

Over the past few years, an upsurge in the incidence of cerebral ischemia (CI) has been observed which is posing increasingly serious threat to public health [20]. It is a hotspot and challenge in modern clinical research to deeply understand the pathogenesis of CI and find a solution for treating it from molecular perspectives [21]. The protective effect of senkyunolide H on cranial nerve has been justified in previous studies [22], but its clinical application has far to go.

In this study, we have initially overcome the technical difficulties in the future clinical application of SH through nanotechnology, which may be a huge breakthrough in the clinical treatment of CI. Our study firstly established rat models with CI and compared the neurological deficit score and NES and S-100*β* between CI rats and normal control group. The results showed notably increased NDS and NES and S-100*β* in the model group, which fully verified the success of the modeling. Neurologic evaluation is not only an index to judge the success of the model but also provides a certain basis for the study of the pathophysiology, model standardization, and drug intervention. Neuron-specific enolase (NES), one enolase implicated in glycolytic pathway, shows the highest activity in brain cells. When brain tissue is damaged, the permeability of tissues and blood vessels will increase, while NES will be released into other tissues in large quantities, causing a higher NES concentration [23]. S-100*β* is an acidic calcium-binding protein, with a high specific response to brain injury and a high association with nervous system diseases [24]. The responses of NES and S-100*β* to nerve injury have been verified in many previous studies [25, 26]. After determined the peak areas under different concentrations of SH-loaded nanoparticle solutions, the results showed that SH-loaded nanoparticles at 10-50 *μ*g/mL had a good reaction effect, which is consistent with the study by Xiong et al. [27] on SH-loaded nanoparticles. Subsequently, we found the size of SH-loaded nanoparticles in the range of 80-120 nm, and that of brain capillary size is approximately 100 nm [28], which also confirms that SH loaded nanoparticles can directly act on brain tissue through brain capillary and blood-brain barrier, thus improving the drug use efficiency.

The article "Senkyunolide H Affects Cerebral Ischemic Injury through Regulation on Autophagy of Neuronal Cells via P13K/AKT/mTOR Signaling Pathway" was retracted in 2023. Reasons: unreliable results or conclusions; concerns about the data; concerns about the peer review; concerns about the citations.

Then, we administered SH-loaded nanoparticles to the CI rats. As a result, the rats showed a decrease in NDS and NES and S-100*β*, which indicates that the nerve injury of rats with CI was alleviated greatly under the intervention of SH-loaded nanoparticles. Earlier studies have also demonstrated the good efficacy of SH on nervous system diseases such as glioma and migraine [29, 30]. It can be due to the following reasons: SH can suppress the induction process of the decrease of erythrocyte deformability index and orientation index by concanavalin A, during which the erythrocyte deformability declines, and it is thus unable to enter the brain tissue through capillaries for blood circulation, finally creating the situation for the first step of cerebral embolism [31]. Then, groups of red blood cells gather and pile up at the blood-brain barrier to form thrombus, which causes both ischemic injury and hypoxia reaction of brain tissue [32]. At the same time, the results of this study showed that the above results can be verified by comparing the brain water content of rats in each group. With the increase of blood-brain barrier permeability, capillary hypoxia edema and brain water content increased [33]. Therefore, the decrease of brain tissue water content indicates that SH has a strong effect on improving brain tissue microenvironment.

For further understanding the mechanism of SH on CI, we investigated the apoptosis and autophagy of neuronal cells (NCs) in the three groups. The results showed that the apoptosis and autophagy of NCs were obviously suppressed after SH intervened, suggesting that the impact of SH on CI might be due to regulation of autophagy of NCs. Beclin-1 and LC3, the most classical autophagy markers, increase with the increase of autophagy in cells [34]. It is precisely because of the acceleration of autophagy that the apoptosis of NCs increases; so, irreversible nerve injury is likely to occur during CI [35]. Moreover, according to one earlier study [36], SH can regulate autophagy of myocardial ischemic cells, which also verifies our results. Finally, we quantified P13K, AKT, and mTOR in brain tissue and found that under intervention with SH, all the three decreased, suggesting the inhibition of P13K/AKT/mTOR pathway. As a classic pathway, it is frequently studied in brain nerve injury diseases [37, 38]. It can mediate the activation of fibroblast growth factor, vascular endothelial growth factor, human growth factor, angiopoietin I, and other substances that stimulate blood and vascular activity and thus promote the development of thrombosis [39]. This study has confirmed that SH-loaded nanoparticles can impact NCs with CI through suppressing P13K/AKT/mTOR signaling pathway.

The article "Senkyunolide H Affects Cerebral Ischemic Injury through Regulation on Autophagy of Neuronal Cells via P13K/AKT/mTOR Signaling Pathway" was retracted in 2023. Reasons: unreliable results or conclusions; concerns about the data; concerns about the peer review; concerns about the citations.

## 5. Conclusion

In this study, we loaded the SH in lipid nanoparticles and successfully obtained SH-loaded nanoparticles with 80-120 nm size in good shape and size distribution uniformity. The intervention of SH-loaded nanoparticles in CI rats can significantly alleviate the nerve injury of CI rats and decrease the apoptosis of the neuronal cells. Meanwhile, the SH-loaded nanoparticles could suppress the autophagy of NCs by medicating P13K/AKT/mTOR signaling pathway and lower apoptosis. Above all, SH-loaded nanoparticle can act as a promising strategy for delivery SH to brain areas, which can be an effective and promising method for treating CI.

## Figures and Tables

**Figure 1:** Flowchart of the presented study.

**Figure 2:** Modeling results. (a) Nerve defect score of the model group compared with the control group. (b) NES concentration of the model group compared with the control group. (c) S-100*β* concentration of the model group compared with the control group. ^∗^ represents *P* < 0.05.

**Figure 3:** Preparation results of SH-loaded nanoparticles. (a) Peak area of SH-loaded nanoparticles solutions. (b) Standard curve.

**Figure 4:** Characterization of SH-loaded nanoparticles. (a) Morphology of SH-loaded nanoparticles visualized under electron microscope. (b) Size distribution of SH-loaded nanoparticles analyzed with PS potentiometer.

The article "Senkyunolide H Affects Cerebral Ischemic Injury through Regulation on Autophagy of Neuronal Cells via P13K/AKT/mTOR Signaling Pathway" was retracted in 2023. Reasons: unreliable results or conclusions; concerns about the data; concerns about the peer review; concerns about the citations.

**Figure 5:** Impact of SH-loaded nanoparticles on NDS of rats compared with the model group and control group. ^∗^ represents *P* value less than 0.05.

**Figure 6:** Impact of SH-loaded nanoparticles on nerve injury compared with the model group and control group. (a) NES concentration of the SH group compared with the model group and control group. (b) S-100*β* concentration of the SH group compared with the model group and control group. (c) BTWC of the SH group compared with the model group and control group. ^∗^ represents *P* value<0.05.

**Figure 7:** Impact of SH-loaded nanoparticles on neuronal apoptosis. (a) Neuronal apoptosis of the SH group compared with the model group and control group. (b) Bax and Bcl-2 proteins of the SH group compared with the model group and control group. ^∗^*P* < 0.05.

**Figure 8:** Impact of SH-loaded nanoparticles on autophagy of NCs compared with the control group and model group.

**Figure 9:** Impact of SH-loaded nanoparticles on P13K/AKT/mTOR pathway in the SH group compared with control and model groups.

## Data Availability

The labeled dataset used to support the findings of this study are available from the corresponding author upon request.
